# Expression and Clinical Significance of *CMTM6* and *PD-L1* in Triple-Negative Breast Cancer

**DOI:** 10.1155/2022/8118909

**Published:** 2022-07-07

**Authors:** Shuai Shi, Hong-Yan Ma, Yin-zhou Sang, Ying-Bo Ju, Xiao-Yun Liu, Zhi-Gang Zhang

**Affiliations:** Department of Pathology, Cangzhou People's Hospital, Cangzhou 061000, China

## Abstract

The CKLF-like MARVEL transmembrane domain containing 6 (*CMTM6*) plays an extremely important role of the programed death receptor ligand-1 (*PD-L1*) protein. Our study is aimed at investigating the expression of *CMTM6* and *PD-L1* proteins in triple-negative breast cancer and their correlation with the clinical pathological data of patients. We selected 89 cases of triple-negative breast cancer and 62 cases of normal breast tissue specimens. Immunohistochemical methods were used to detect the expression levels of *CMTM6* and *PD-L1* and to carefully study differences in their expression. The expression of *CMTM6* and *PD-L1* in TNBC was higher than that in normal breast tissue, and the expression of the two was positively correlated (*p* < 0.05). In TNBC, *CMTM6* expression is positively correlated with tumor size, lymph node metastasis, Ki67 proliferation index, and TNM stage (*p* < 0.05). *PD-L1* expression is positively correlated with tumor size, lymph node metastasis, Ki67 proliferation index, TNM stage, and vascular infiltration (*p* < 0.05). Kaplan-Meier analysis showed that the positive expression of *CMTM6* and *PD-L1* had no correlation with the survival rate of patients (*p* > 0.05). According to KM-plotter, we found that a higher CMTM6 expression was positively related with relapse-free survival rate of patients (*p* < 0.05). A higher PD-L1 expression was positively correlated with relapse-free, overall, and distant metastasis survival rate of patients (*p* < 0.05). In timer database, we found a positive correlation between the expression of CMTM6 and PD-L1 in triple-negative breast cancer. Both *CMTM6* and *PD-L1* are highly expressed in TNBC, and their expressions are positively related. In the future, the two gene might become targets for the treatment of TNBC, providing a basis of clinical treatment of TNBC.

## 1. Introduction

Breast cancer is a common malignant tumor for women. As the incidence of breast cancer has gradually increased, it has made an important threat to women's health [1]. Breast cancer is divided into four subtypes based on receptor types: luminal A, luminal B, Her2 +, and triple-negative. Triple-negative breast cancer (TNBC) has the characteristics of high transfer rate, low degree of differentiation, poor treatment, and low survival rate. Chemokine plays an important role in the process of tumors and autoimmune diseases [2]. Triple-negative breast cancer is a clinicopathological classification based on the results of immunohistochemistry. The basel-like group of triple-negative breast cancer and molecular typing (PAM50) has a high degree of overlap [3]. At present, the standard treatment of TNBC is mainly chemotherapy, and targeted therapy and immunotherapy are constantly being explored [4]. Peking University first discovered 8 new genes of the chemokine family. It has the characteristics of MARVEL structures, so the chemokine-containing factor super family 1-8 (CKLF-like MARVEL transmembrane domain containing 1-8 (CMTM1-8)) is named MARVEL transmembrane structure [5]. Chemokine-like factor super family member 6 (*CMTM6*) is one of the members of the CMTM family. *CMTM6* is located in chromosome P22, with 183 amino acids, and molecular weight is 20.4 kD. *CMTM6* is widely expressed in normal human tissues, mainly located on the cell membrane, and participates in epigenetic regulation and tumorigenesis [6]. Studies have shown that *CMTM6* is abnormally expressed in colorectal cancer, lung cancer, and glioma [7–9].

*PD-L1* is also known as CD274 and belongs to the B7 family. The *PD-L1* is the type I transmembrane protein, the molecular weight is 33 kD, and the PD-1 gene encoding chemical assembly instruction inside of living things of human 9 chromosome is encoded, which is the ligand of PD1. When PD1 binds to *PD-L1*, it inhibits the activation of tumor antigen-specific T cells, thereby downregulating the expression of antiapoptotic molecules and proinflammatory factors [10]. The combination of PD-1 and *PD-L1* can affect the cell cycle, make tumor cells evade the body's immune killing, and ultimately lead to the occurrence and development of tumors [11]. There are studies targeting programmed cell death ligand 1 (PD-L1) with monoclonal antibodies (mAbs) such as atezolizumab to treat various tumors. Molecular mechanisms of response to atezolizumab use the PD-L1-expressing human TNBC cell line MDA-MB-231. Atezolizumab downregulates genes that promote cell migration/invasion and metastasis, epithelial-mesenchymal transition (EMT), cell growth/proliferation/survival, and hypoxia. Conversely, genes related to apoptosis and DNA repair were upregulated after atezolizumab treatment. The findings suggest that monoclonal antibodies (mAbs) such as atezolizumab target programmed cell death ligand 1 (PD-L1) to inhibit TNBC molecular mechanisms/signaling pathways provide new insights [12]. Previous studies have shown that *CMTM6* can be used as a key regulator of *PD-L1* in a variety of tumor cells, binds to *PD-L1* and maintains its stable expression of the cell surface, and does not make *PD-L1* lysosome-mediated degradation target [13, 14]. The deletion of the *CMTM6* gene will cause the degradation of *PD-L1* protein and reduce its expression of the surface of tumor cells. The specific binding of *CMTM6* and *PD-L1* can maintain the recycling of the *PD-L1*/*CMTM6* protein complex in the inclusion body and protect the *PD-L1* protein from being recognized and degraded by lysosomes and ultimately maintain the high expression of *PD-L1* [15].

In our study, we detected the expression of *CMTM6* and *PD-L1* in triple-negative breast cancer, analyzed their relationship with clinicopathological characteristics, and explored the clinical significance of *CMTM6* and *PD-L1* in triple-negative breast cancer.

## 2. Material and Methods

### 2.1. Tissue Samples

Collected paraffin specimens of triple-negative breast cancer (*n* = 89) and normal breast tissue (*n* = 62) are from Cangzhou People's Hospital. The patients were 26-81 years old, with an average age of 51.0 years. During the preoperative interview, we provided written informed consent for the patient to describe the use of his tissue. This study was reviewed by the Ethics Committee of Cangzhou People's Hospital (approval number: J2022-001(0121)). All cases did not undergo radiotherapy, chemotherapy, and biological therapy before surgery. All specimens were histologically diagnosed by two pathologists, including 38 histological grade I cases and 51 histological grade II-III cases. According to the American Joint Committee on Cancer (AJCC), triple-negative breast cancer was classified by TNM, including 73 cases of stage I and 16 cases of stages II-III.

### 2.2. Immunohistochemistry

All specimens were fixed in neutral formaldehyde solution at 37°C, embedded in paraffin, sectioned at 4 *μ*m, and stained with HE. After dewaxing and hydration, the tissue chip was repaired under high pressure, and the primary antibody was added dropwise for 15 min and then incubated at 4°C overnight. After washing with PBS, the secondary antibody was added and incubated at room temperature for 17 min. The bag used for the primary antibody incubation is transparent and sealed. The primary antibody is rabbit *CMTM6* (Abcam; 1 : 100; ab264067) and PD-L1 (Abcam; 1 : 100; ab205921). Then, anti-rabbit antibodies conjugated to HRP (Abcam, 1 : 200, ab996979) were subjected to incubation as the secondary antibody. Use 3, 3′-diaminobenzidine to observe the binding sites and then counterstained with Mayer's hematoxylin. Both *CMTM6* and *PD-L1* proteins are located on the cell membrane.

Two independent observers score the slices separately (Shi S and Ma HY). The inconsistent data were confirmed by both persons until final agreements were reached. The expression positivity was graded and counted as follows: 0 = negative, 1 = 1-50%, 2 = 50-74%, and 3 ≥ 75%. The staining intensity score was graded as follows: 1 = weak, 2 = intermediate, and 3 = strong. The scores for CMTM6 [16] and PD-L1 [17] positivity and staining intensity were multiplied to obtain a final score, which determines their expression as (− = 0 − 2; + = 3-9).

### 2.3. Kaplan-Meier Plotter and TIMER Analysis

The prognosis of CMTM6 and PD-L1 was analyzed using KM-plotter (http://www.kmplot.com) and TIMER (https://cistrome.shinyapps.io/timer/) database, and the correlation of CMTM6 and PD-L1 in triple-negative breast cancer was analyzed.

### 2.4. Statistical Analysis

The results are analyzed by the SPSS 17.0 software (SPSS). The chi-square test was used to compare the expression differences between TNBC and normal breast tissues. Fisher's exact test was used to analyze the correlation between *CMTM6* and *PD-L1* in TNBC. Kaplan-Meier method was used for survival analysis, and COX risk regression models were used for univariate multivariate analysis. *p* value of < 0.05 was considered statistically significant.

## 3. Results

### 3.1. Expression of CMTM6 and PD-L1 in TNBC and Normal Breast Tissue

As shown in Figures 1(a) and 1(d), we performed HE staining on triple-negative breast cancer tissue and normal breast tissue. The results of immunohistochemistry showed that *CMTM6* and *PD-L1* proteins were located on the cell membrane, and their expression in TNBC (Figures 1(e) and 1(f)) was higher than that in normal breast tissues (Figures 1(b) and 1(c)). The positive rates of *CMTM6* in TNBC and normal breast tissue were 56.2% (50/89) and 16.1% (10/62), respectively (*p* < 0.05, Table 1). *PD-L1* expression was detected in 29.2% (26/89) of TNBC and 8.1% (5/62) of normal breast tissue (*p* < 0.05, Table 1). In TNBC, the expression of *CMTM6* and *PD-L1* was positively correlated (*p* < 0.05, Table 2).

### 3.2. Association of CMTM6 and PD-L1 Expression with the Clinicopathological Parameters of TNBC

We collected the clinicopathological data of 89 patients with TNBC, including patient age, tumor size, TNM staging, histological grade, vascular infiltration, nerve invasion, lymph node status, TP53, Ki67, and distant metastasis. As shown in Table 3, *CMTM6* expression is positively correlated with tumor size, lymph node metastasis, Ki67 proliferation index, and TNM staging (*p* < 0.05). *PD-L1* expression is positively correlated with tumor size, lymph node metastasis, Ki67 proliferation index, TNM staging, and vascular infiltration (*p* < 0.05). With the increase of TNM stage, the expression of CMTM6 and PD-L1 in triple-negative breast cancer patients also increased.

### 3.3. Relationship between CMTM6 and PD-L1 Expression and Prognosis of TNBC

Kaplan-Meier analysis showed that the positive expression of *CMTM6* and *PD-L1* had no correlation with the survival rate of patients (Figures 2(a) and 2(b), *p* > 0.05). During the cox survival analysis, due to the small number of samples and the short follow-up time of patients, no prognostic indicators and independent risk factors were found to affect the prognosis of patients with triple-negative breast cancer (*p* > 0.05, Tables 4 and 5). According to KM-plotter, we found that a higher CMTM6 expression was positively related with relapse-free survival rate of patients (Figure 3(a)). A higher PD-L1 (CD274) expression was positively correlated with relapse-free, overall, and distant metastasis survival rate of patients (Figure 3(b)). In TIMER database, we found a positive correlation between the expression of CMTM6 and PD-L1 in triple-negative breast cancer(Figure 3(c)).

## 4. Discussion

Breast cancer is a common malignant tumor that endangers women's health. With the advancement of medicine, the early diagnosis and treatment of breast cancer have made great progress, but for advanced patients, radiotherapy and chemotherapy are still the main treatment methods. Studies have shown that the overall survival rate of patients with triple-negative breast cancer is significantly lower than that of patients with non-triple-negative breast cancer [18]. In recent years, immunotherapy has been widely used in cancer treatment in recent years. In recent years, immunotherapy had been widely used in tumor treatment. Compared with traditional radiotherapy and chemotherapy, immunotherapy can target tumors, thereby inhibiting immune escape pathways and ultimately inhibiting tumor growth. Therefore, finding new immunotherapy targets is of great significance for the early diagnosis, treatment, and prognosis of breast cancer patients.

As a member of the CMTM family, *CMTM6* is widely expressed in human tissues, mainly on cell membranes. Studies have found that the high expression of *CMTM6* can negatively regulate T cells to kill tumors, thereby participating in the occurrence and development of tumors [19]. Previous studies have shown that *CMTM6* is elevated in colorectal cancer, non-small-cell lung cancer, glioma, melanoma, and other tissues [7–9, 14, 20]. Our study found that *CMTM6* is also highly expressed in triple-negative breast cancer. Yang et al. found that the expression of *CMTM6* was correlated with the pathological type of breast cancer patients and HER2 positivity. Breast cancer pathological classification, TNM stage, triple-negative breast cancer, and high expression of *CMTM6* could be used as independent risk factors to judge the prognosis of patients [21]. Our research in triple-negative breast cancer showed that *CMTM6* was not an independent risk factor for triple-negative breast cancer. The paradoxical results might be due to the selection of samples and the number of samples, the small number of samples in our hospital, and the short follow-up time for patients. On the contrary, the expression of *CMTM6* in hepatocellular carcinoma and esophageal cancer tissues is lower than that in normal tissues, which indicates that *CMTM6* expression is different in different tissues [20, 22]. This difference determines the biological characteristics of different tumors. The specific reasons need to be further explored.

The PD-1/*PD-L1* signaling pathway is a pair of costimulatory molecules in the process of T cell immune response. It induces antigen-specific T cell apoptosis by negatively regulating T lymphocyte activation, proliferation, and effector functions and exerts an immunosuppressive effect. Monoclonal antibodies targeting the PD-1/PD-Ll pathway had been developed into tumor immunotherapy by improving the function of T lymphocytes, and its clinical trials had also shown exciting effects. As the ligand of PD-1, *PD-L1* is mainly expressed on mature immune cells and is highly expressed on the surface of a variety of tumor cells [23]. The expression of *PD-L1* in melanoma, non-small-cell lung cancer, and gastric cancer was higher than that in adjacent tissues, and survival analysis suggests that *PD-L1* might be a predictor of tumor prognosis [24–26]. Studies had shown that the expression of *PD-L1* protein and mRNA in triple-negative breast cancer was higher than that of adjacent tissues, and *PD-L1* expression was positively correlated with lymph node metastasis, ki67 proliferation index, and histological grade [27, 28]. Our research showed that the expression of *PD-L1* in TNBC was higher than that in normal breast tissue. *PD-L1* expression was positively correlated with tumor size, lymph node metastasis, Ki67 proliferation index, TNM stage, and vascular infiltration.

Burr et al. [13] found that the deletion of the *CMTM6* gene can cause the degradation of *PD-L1* protein and reduce its expression on the cell surface. The specific binding of *CMTM6* and *PD-L1* can maintain the recycling of the *PD-L1*/*CMTM6* complex in the inclusion body, thereby protecting the *PD-L1* protein from being recognized and degraded by lysosomes, and maintaining the high expression of the *PD-L1* protein. *PD-L1* can regulate the stability of RNA, but when the interaction between *CMTM6* and *PD-L1* is eliminated, the stability of *PD-L1* is destroyed, and the binding of *PD-L1* to the RNA of the target gene is also destroyed, eventually leading to degradation of target RNA [29]. The stability regulation of *CMTM6*/*PD-L1* on gene group RNA indirectly proves that *CMTM6*/*PD-L1* plays a more important role in tumor development and the survival status of tumor cells themselves.

## 5. Conclusions

In conclusion, upregulated expression of *CMTM6* and *PD-L1* may play a role in the occurrence and development of TNBC. It might be considered a good biomarker to indicate the aggressiveness of TNBCs. In the future, whether *CMTM6* and *PD-L1* can be used as prognostic indicators of triple-negative breast cancer requires a large number of samples to verify. The study of *CMTM6* and *PD-L1* in the pathogenesis of triple-negative breast cancer requires further research.

## Figures and Tables

**Figure 1:** *CMTM6* and *PD-L1* expression in TNBC. HE staining on triple-negative breast cancer tissue and normal breast tissue (a, d). The expression of *CMTM6* and *PD-L1* in normal breast tissues (b, c). The expression of *CMTM6* and *PD-L1* in TNBC (e, f).

**Figure 2:** Relationship between *CMTM6* and *PD-L1* expression and prognosis of TNBC. Kaplan-Meier analysis of overall survival associated with *CMTM6* (a) and *PD-L1* (b).

**Figure 3:** Correlation and prognostic significance of CMTM6 and PD-L1 expression in triple-negative breast cancer. According to KM-plotter, we found that a higher CMTM6 expression was positively related with relapse-free survival rate of patients (a). A higher PD-L1 expression was positively correlated with relapse-free, overall, and distant metastasis survival rate of patients (b). In TIMER database, we found a positive correlation between the expression of CMTM6 and PD-L1 in triple-negative breast cancer (c).

**Table 1:** CMTM6 and PD-L1 expression in normal tissue and TNBC.

Groups	*n*	CMTM6 expression			PD-L1 expression		
		—	+	PR (%)	—	+	PR (%)
Normal	62	52	10	16.1	57	5	8.1
Cancer	89	39	50	56.2^∗^	63	26	29.2^∗^

PR: positive rate. ^∗^*p* < 0.01.

**Table 2:** Correlation analysis of CMTM6 and PD-L1 in TNBC.

CMTM6	PD-L1		Total	*p* value
	Positive	Negative		
Positive	20	30	50	0.01
Negative	6	33	39	
Total	26	63	89	

**Table 3:** Relationship between expression of CMTM6 and PD-L1 protein and clinicopathological features of TNBC.

Clinicopathological features	*n*	Protein expression							
		CMTM6				PD-L1			
		—	+	PR (%)	*p* value	—	+	PR (%)	*p* value
Age									
≤50	36	14	22	61.1	0.147	24	12	33.3	0.181
>50	53	25	28	52.8		39	14	26.4	
Size									
<3	50	25	25	50.0	0.043	38	12	24.0	0.022
≥3	39	14	25	64.1		25	14	35.9	
Lymph node metastasis									
-	54	27	28	51.9	0.028	47	8	14.8	<0.001
+	34	12	22	64.7		16	18	52.9	
Distant metastasis									
-	81	36	45	55.6	0.298	60	21	25.9	0.273
+	8	3	5	62.5		3	5	62.5	
TNM stage									
I	73	34	39	53.4	0.003	57	16	21.9	0.039
II-III	16	5	11	68.8		6	10	62.5	
Histological grade									
I	38	15	23	60.5	0.187	31	7	18.4	<0.001
II-III	51	24	27	52.9		32	19	37.3	
Vascular infiltration									
-	52	25	27	51.9	0.091	41	11	21.2	0.001
+	37	14	23	62.2		22	15	40.5	
Nerve invasion									
-	75	34	41	54.7	0.076	53	22	29.3	0.909
+	14	5	9	64.3		10	4	28.6	
TP53									
-	23	11	12	52.2	0.531	17	6	26.1	0.429
+	66	28	38	57.6		46	20	30.3	
Ki67									
-	10	8	2	20.0	<0.001	10	0	0.0	<0.001
+	79	31	48	60.8		53	26	32.9	

PR: positive rate.

**Table 4:** Univariate analysis of prognostic risk factors in the patients with TNBC.

Characteristics	CMTM6		PD-L1	
	Relative risk (95% CI)	*p* value	Relative risk (95% CI)	*p* value
Size				
<3	0.698 (0.062-7.835)	0.771	0.202 (0.018-2.262)	0.194
≥3				
Age(years)				
<60	0.680 (0.060-7.694)	0.755	0.235 (0.020-2.747)	0.248
≥60				
Lymph node metastasis				
-	0.897 (0.081-9.893)	0.929	0.530 (0.048-5.853)	0.605
+				
Distant metastasis				
-	0.752 (0.068-8.314)	0.816	0.442 (0.035-5.541)	0.527
+				
TNM stage				
I	0.907 (0.081-10.118)	0.937	0.444 (0.035-5.716)	0.534
II-III				
Histological grade				
I	0.729 (0.065-8.130)	0.797	0.186 (0.016-2.147)	0.178
II-III				
Vascular infiltration				
-	0.790 (0.070-8.945)	0.849	0.241 (0.021-2.808)	0.256
+				
Nerve invasion				
-	0.551 (0.048-6.352)	0.632	0.172 (0.015-1.922)	0.153
+				
TP53				
-	0.608 (0.055-6.725)	0.685	0.202 (0.018-2.228)	0.191
+				
Ki67				
-	0.822 (0.074-9.085)	0.873	0.248 (0.022-2.734)	0.255
+				

CI: confidence interval; TNM: tumor-node-metastasis.

**Table 5:** Multivariate analysis of clinicopathological variables for the survival of the patients with TNBC.

Clinicopathological parameters	*p*	*p*
CMTM6/PD-L1 expression (+)	0.982	0.827
Size (≥3)	0.814	0.767
Age (≥60 years)	0.966	0.929
Lymph node metastasis (+)	0.937	0.837
Distant metastasis (+)	0.719	0.632
TNM staging (III–IV)	0.999	0.954
Histological grade (III–IV)	0.398	0.529
Vascular infiltration (+)	0.998	0.982
Nerve invasion (+)	0.822	0.733
TP53 (+)	0.997	0.943
Ki67 (+)	0.934	0.961

CI: confidence interval; TNM: tumor-node-metastasis.

## Data Availability

The data used to support the findings of this study are included within the article.
